The article "Relationships between 25-Hydroxyvitamin D and Nocturnal Enuresis in Five- to Seven-Year-Old Children" was published in 2014. Journal: PLoS One.

# Relationships between 25-Hydroxyvitamin D and Nocturnal Enuresis in Five- to Seven-Year-Old Children

**DOI:** 10.1371/journal.pone.0099316

**Published:** 2014-06-09

**Authors:** Luanluan Li, Huafei Zhou, Xin Yang, Li Zhao, Xiaodan Yu

**Affiliations:** 1 MOE-Shanghai Key Lab of Children's Environmental Health, Shanghai Institute for Pediatric Research, Xinhua Hospital affiliated to Shanghai Jiao Tong University School of Medicine, Shanghai, China; 2 Taizhou Hospital at Luqiao, Zhejiang Province, China; University of Bari Aldo Moro, Italy

## Abstract

**Background:**

Vitamin D has been recognized to contribute to various physiological processes. However, no study has investigated serum 25-hydroxyvitamin D [25(OH)D] concentrations in children with nocturnal enuresis (NE) in the English literature.

**Objective:**

In the present study, serum 25(OH)D concentrations were measured in five- to seven-year-old children with NE and compared with those in non-enuretic children to investigate whether there was any relationship between 25(OH)D and NE as the first time in the literature.

**Design:**

Two hundred forty-seven five- to seven-year-old children were recruited from Taizhou, Zhejiang Province, China. Serum 25(OH)D concentrations were measured, and the structured questionnaire was administered to the parents of all children. Low 25(OH)D was defined as serum 25(OH)D concentrations below 20 ng/ml.

**Results:**

The prevalence of NE was 7.3% in the group of children with 25(OH)D concentrations that exceeded 20 ng/ml; this prevalence was much lower than the 17.5% observed in the group of children with 25(OH)D concentrations below 20 ng/ml (p<0.05). After adjusting for potential confounders, serum 25(OH)D (≥20 ng/ml) was significantly associated with NE and represented a protective factor against NE (OR = 0.31, 95%CI = 0.092, 1.0, P<0.05). A nonlinear relationship between 25(OH)D and NE was observed. The prevalence of NE decreased with increasing 25(OH)D concentrations above 19 ng/ml. Additionally, children exhibiting higher frequencies of bedwetting had lower 25(OH)D concentrations [5–7 times/week: 18.3±4.8; 2–4 times/week: 20.9±4.1; 0–1 times/week: 23.6±6.4 (ng/ml), P<0.05)].

**Conclusions:**

Low 25(OH)D was associated with an increased risk of NE in children aged five to seven years.

## Introduction

The major role of vitamin D in the human body is commonly thought to be related to calcium metabolism and bone structure. However, scientific evidence clearly indicates that the biological importance of this vitamin greatly exceeds these aspects. The 25-hydroxyvitamin D [25(OH)D] is the main circulating metabolite of vitamin D, and is considered to be an indicator of vitamin D status in the human body [1]. Low 25(OH)D is considered to play an important role in the development of cardiovascular diseases, metabolic syndrome, type 2 diabetes mellitus, inflammatory and immune abnormalities, and sleep disorders [2]–[4]. To the best of our knowledge, there is no report concerning the relationship between 25(OH)D and nocturnal enuresis (NE) in the English literature.

The article "Relationships between 25-Hydroxyvitamin D and Nocturnal Enuresis in Five- to Seven-Year-Old Children" was published in 2014. Journal: PLoS One.

NE is defined as nighttime bedwetting (≥2times per week) in children five years of age or older [5] and is the most common voiding problem in pediatric population. The prevalence of NE in children worldwide has been reported to range from 1.4% to 28% depending on the definition of enuresis, children's ages, and cultural differences [6]–[7]. Due to its high prevalence, NE has remained a focus of extensive scientific research over the past few decades. The etiology of NE has been widely debated but currently remains unclear. The commonly established causes of NE are arousal dysfunction and nocturnal polyuria [8]–[9]. Arousal dysfunction is related to sleep disorders [10]. Anatomic evidence and clinical studies suggest that vitamin D may be involved in sleep regulation [4], [11]–[13]. Besides, vitamin D deficiency is associated with the severity of obstructive sleep apnea (OSA) [14]–[19], and nocturnal polyuria is one of the main adverse outcomes of OSA [20]. Moreover, vitamin D deficiency could directly lead to excessive urine production [21]. Therefore, we propose the hypothesis that there is some connection between NE and vitamin D.

In the present study, serum 25(OH)D concentrations were measured in five- to seven-year-old children with NE and compared with those in non-enuretic children to investigate any potential relationship between 25(OH)D and NE, and for the first time in the literature, to explore the possibility that a threshold serum 25(OH)D concentration in relation to NE exists in young children.

## Subjects and Methods

### Subjects

From November 2012 to March 2013, 247 children were recruited from five kindergartens in Taizhou, Zhejiang Province, China. These children's ages ranged from 5 to 7 years old. 134 boys (54.3%) and 113 girls (45.7%) participated. Exclusion criteria included the following: 1) any medication or treatment related to nocturnal enuresis; 2) supplemental vitamin D intake >400 IU/d; 3) subjects with age <5 years old. Participation in the study was voluntary, and written informed consent was obtained from children's parents. This study was approved by the Ethics Committee of Shanghai Jiao Tong School of Medicine, China.

### Questionnaires

A face-to-face interview with the parents was conducted by a trained doctor using a structured questionnaire. The information collected included the child's age, gender, gestational age, birth weight, maternal education, paternal education, and family income. Nighttime bedwetting and its severity were also recorded. The frequencies of bedwetting were graded as “occasionally” (0–1 times per week), “frequently” (2–4 times per week), and “almost always” (5–7 times per week). In this study, NE was defined as nighttime bedwetting (≥2times per week) in children five years of age or older [5].

The article "Relationships between 25-Hydroxyvitamin D and Nocturnal Enuresis in Five- to Seven-Year-Old Children" was published in 2014. Journal: PLoS One.

### Serum 25(OH)D measurement

Fasting venous blood samples from all participants were collected in the early morning. Serum was separated and stored in lightproof containers at −20°C until the samples were assayed for vitamin D metabolites. We used the sensitive liquid chromatographytandem mass spectrometry (LC-MS/MS) analytical method to detect serum 25(OH)D, as reported by van den Ouweland JM et al. [22]. The serum samples (100 µl) were deproteinised and precipitated using methanol, acetonitrile, zinc sulfate, and internal standards that included deuterated 25(OH)D_2_ and 25(OH)D_3_ (Sigma USA). Chromatographic separations were achieved on an Agilent Poroshell 120 EC-C18(50×2.1 mm, 2.7 µm) column with a gradient of water (containing 0.1% formic acid) and methanol as the mobile phase at a flow rate of 0.5 mL/min. Multiple reaction monitoring (MRM) of the analytes was performed under electrospray ionization (ESI) in the positive mode at m/z 401.3→383.2 and 401.3→159.1 for 25(OH)D_3_, m/z 413.3→395.3 and 413.3→355.2 for 25(OH)D_2_, and m/z 404.3→386.3 and 416.4.3→398.3 for d_3_-25(OH)D_3_ and d_3_-25(OH)D_2_, respectively. Low 25(OH)D was defined as serum 25(OH)D concentrations <20 ng/ml [23]–[25].

### Statistical analyses

Serum 25(OH)D concentrations analyzed in our study were normally distributed. We first performed a univariate analysis to examine group differences in NE (Table 1) and then used multiple linear regression to estimate the independent relationship between 25(OH)D and NE after adjusting for potential confounders (Table 2). Next, we constructed a generalized additive model to explore the relationship between 25(OH)D and NE via a smoothing plot (Figure 1). We further applied a two-piecewise linear regression model to examine the threshold effect of 25(OH)D on NE according to the smoothing plot (Table 3). The inflection of 25(OH)D concentrations (i.e., the point at which the relationship between 25(OH)D and NE began to change shape and become prominent) was determined using a trial method. This trial method involved moving the trial inflection point along a pre-defined interval and detecting the inflection point that produced the maximum model likelihood. Finally, analysis of variance was used to examine the effect of 25(OH)D on the frequency of bedwetting (Figure 2). All analyses were performed using Empower(R) (version 2.13.9, X&Y solutions, Inc., Boston, MA) and R (version 2.15.3, Robert Gentleman and Ross Ihaka, Auckland, New Zealand).

The article "Relationships between 25-Hydroxyvitamin D and Nocturnal Enuresis in Five- to Seven-Year-Old Children" was published in 2014. Journal: PLoS One.

**Figure 1:** The Relationship between 25(OH)D and nocturnal enuresis. A nonlinear relationship between serum 25(OH)D concentrations and nocturnal enuresis was observed after adjusting for gender, age, gestational age, birth weight, maternal education, paternal education, and family income. A threshold for 25(OH)D of 19 ng/ml existed for nocturnal enuresis. 25(OH)D, 25-hydroxyvitamin D.

**Figure 2:** The effect of 25(OH)D on the frequency of bedwetting. Serum 25(OH)D concentrations (mean ± SD): 5–7 times/week: 18.3±4.8(ng/ml); 2–4 times/week: 20.9±4.1(ng/ml); 0–1 times/week: 23.6±6.4 (ng/ml). Compared to the 5–7 times/week and 2–4 times/week groups, the concentrations of 25(OH)D in the 0–1 times/week group were much higher (P<0.05). 25(OH)D, 25-hydroxyvitamin D.

**Table 1:** Effects of risk factors on nocturnal enuresis (n = 247).*

		Nocturnal Enuresis	
	%	%	p-value
**25(OH)D dichotomous**			
<P50(22.2 ng/ml)	50	17.0	<0.05
≥P50(22.2 ng/ml)	50	6.8	
**Low 25(OH)D (<20 ng/ml)**			
Yes	29.9	17.5	<0.05
No	70.1	7.3	
**Gender**			
male	54.3	16.0	>0.05
female	45.7	8.3	
**Age**			
5 years	33.2	15.4	>0.05
6 years	47.0	12.2	
7 years	19.8	8.6	
**Gestational age**			
Preterm infant	8.9	20.0	>0.05
Term infant	91.1	11.6	
**Low birth weight**			
No	98.0	13.5	>0.05
Yes	2.0	0	
**Maternal education**			
Primary school	23.2	17.9	>0.05
Middle school	58.5	13.5	
High school	13.7	6.5	
Bachelor degree or higher	4.6	0	
**Paternal education**			
Primary school	14.1	19.2	>0.05
Middle school	64.3	13.6	
High school	18.3	7.9	
Bachelor degree or higher	3.3	0	
**Family incomes (Yuan/m/person)**			
≤1000	21.2	28.6	>0.05
1000–2000	29.1	7.6	
2000–5000	22.2	14.8	
≥5000	27.5	7.7	

25(OH)D, 25-hydroxyvitamin D.

*Determined by univariate analysis.

**Table 2:** Adjusted effect of 25(OH)D on nocturnal enuresis.

	Nocturnal Enuresis	
	β/OR (95%CI) P-value	
	Unadjusted*	Adjusted#
**25(OH)D**	0.94 (0.87, 1.0)>0.05†	0.9 (0.8, 1.0)<0.05†
**25(OH)D**		
<20(ng/ml)	1.0	1.0
≥20 (ng/ml)	0.52 (0.21, 1.3)<0.05‡	0.31 (0.092,1.0)<0.05‡

β, regression coefficient; 25(OH)D, 25-hydroxyvitamin D.

*Unadjusted and analyzed by using liner regression.

# Adjusted for gender, age, gestational age, birth weight, maternal education, paternal education, and family income by using multiple linear regression.

† Unadjusted β, 0.94; adjusted β, 0.9.

‡ Unadjusted OR, 0.52; adjusted OR, 0.31.

The article "Relationships between 25-Hydroxyvitamin D and Nocturnal Enuresis in Five- to Seven-Year-Old Children" was published in 2014. Journal: PLoS One.

**Table 3:** Threshold effect analysis of 25(OH)D on nocturnal enuresis.*

Inflection point of 25(OH)D(ng/ml)	Nocturnal Enuresis
	OR (95%CI) p-value
19.0	
<19.0	1.0 (0.77, 1.3) 0.96
≥19.0	0.84 (0.7, 1.0)<0.05

25(OH)D, 25-hydroxyvitamin D.

*Adjusted for gender, age, gestational age, birth weight, maternal education, paternal education, and family income by using piece-wise linear regression.

P values less than 0.05 were considered statistically significant. Moreover, because p values depend on the size of the data set, statistical inferences were assessed using estimation with confidence intervals (CI) and odds ratios (OR). If the 95% CI excluded 1, the difference between the groups was considered significant, and if the 95% CI included one, the difference was considered non-significant at p = 0.05.

## Results

A total of 247 (134 males and 113 females) children aged 5 to 7 years were recruited. Of these children, 8.9% were preterm infants (gestational age<37 weeks) and 2.0% had low birth weights (birth weight<2500 grams). The median serum 25(OH)D concentration was 22.2 ng/ml, which is higher than the recommended concentration (20 ng/ml), and 29.9% of the children had low 25(OH)D concentrations (Table 1).

Table 1 shows the unadjusted associations between 25(OH)D and NE. Serum 25(OH)D concentrations were associated with NE in the dichotomous analyses. The prevalence of NE decreased with the increase across the dichotomous concentrations of 25(OH)D (p<0.05). Compared to the children with 25(OH)D concentrations above 20 ng/ml, the children with 25(OH)D concentrations below 20 ng/ml exhibited a greater risk of NE (p<0.05). Additionally, there was no association between NE and the child's gender, age, gestational age, birth weight, maternal or paternal education level, or family income (p>0.05).

Table 2 shows the adjusted association between 25(OH)D and NE. After adjusting for gender, age, gestational age, birth weight, maternal and paternal education, and family income, serum 25(OH)D concentrations were negatively associated with NE [regression coefficient (β) = 0.9, 95% CI = 0.8, 1.0, p<0.05], and serum 25(OH)D greater than 20 ng/ml represented a protective factor against NE (OR = 0.31, 95% CI = 0.092, 1.0, p<0.05).

There was a nonlinear relationship between serum 25(OH)D and NE after adjusting for confounders (Figure 1). When serum 25(OH)D concentrations were above the inflection point (19 ng/ml), the prevalence of NE decreased with increasing 25(OH)D concentrations (OR = 0.84, 95% CI = 0.7, 1.0, p<0.05) (Table 3).

Figure 2 illustrates that higher frequencies of bedwetting were associated with lower 25(OH)D concentrations [5–7 times/week:18.3±4.8, 2–4 times/week: 20.9±4.1, and 0–1 times/week: 23.6±6.4 (ng/ml),P<0.05)].

The article "Relationships between 25-Hydroxyvitamin D and Nocturnal Enuresis in Five- to Seven-Year-Old Children" was published in 2014. Journal: PLoS One.

## Discussion

In the present study, a statistically significant association was found between serum 25(OH)D and NE. Our data revealed that that children with lower 25(OH)D concentrations were at an increased risk of NE. We searched the medical literature for information about serum 25(OH)D concentrations in enuretic children and were unable to find any studies on this topic. Therefore, we report here, for the first time, a negative relationship between 25(OH)D and NE in 5–7 year-old children.

Vitamin D, apart from its classical effect on the regulation of calcium homeostasis and bone metabolism, has been recognized to contribute to various physiological processes. The effect of vitamin D on NE is associated with its influence on sleep disorders, OSA, and nocturnal polyuria.

NE is a common problem among children. Data have accumulated pointing to an association of sleep disorders with NE in some children, which is consistent with the report of T. Nevéus [26] that states that NE is not only a nocturnal problem but also a disorder of sleep. The parents of children who wet the bed often claim that their children are “deep sleepers”. Children with NE may, however, experience sleep disorders. One recent study of children with NE indicates that the sleep of these children is significantly more fragmented and that these children experience excessive daytime sleepiness [27]. This sleep fragmentation leads to an increased arousal threshold [10], [28], which, in turn, results in the loss of physiologic inhibitory signals to the bladder that have been observed in animal studies [29].

Sleep disorders may play a role in development of NE. Based on this finding, we measured serum 25(OH)D concentrations, effective on sleep patterns, in enuretic children. There is an anatomic evidence for an association between 25(OH)D and sleep patterns, which is supported by the presence of vitamin D receptors in the anterior and posterior hypothalamus, substantia nigra, midbrain central gray, raphe nuclei, and the nuclei reticularis pontis oralis and caudalis [11]. These same areas are thought to play important roles in the initiation and maintenance of sleep. Moreover, clinical studies suggest that vitamin D supplementation for patients with sleep disorders may contribute to significant improvements in sleep quality [4], [12]–[13].

Low 25(OH)D is proposed to contribute to immune dysregulation including inducing a relative elevation of circulating IL-1, IL-2, IL-6, TNFα and NFκB, all of which can result in subjective sleepiness symptoms [30]–[34]. Therefore, it is mechanistically plausible that suboptimal concentrations of 25(OH)D may contribute to poor sleep quality by directly modulating immune-regulating substances [35]. Together, these studies confirm the hypothesis that Low 25(OH)D contributes to sleep disorders, which, in turn, lead to an increase in the risk of NE. However, this hypothesis is still under discussion and need to be confirmed by further studies.

The article "Relationships between 25-Hydroxyvitamin D and Nocturnal Enuresis in Five- to Seven-Year-Old Children" was published in 2014. Journal: PLoS One.

Another possible mechanism involves an interaction between vitamin D deficiency and other disorders, particularly OSA. Vitamin D deficiency is correlated with chronic rhinitis [14], tonsillar hypertrophy [15]–[16], and nonspecific myopathy [17]–[19], all of which are known to increase the risk of OSA. Therefore, Low 25(OH)D represents a plausible factor that could lead to more severe OSA.

Sleep research has documented that NE is related to OSA in children [36]–[37]. Nocturnal polyuria is considered to be a characteristic of OSA [20]. Patients with OSA excrete large amounts of urine overnight [20], probably because of increased secretion of atrial natriuretic peptide (ANP), which is released from the heart in response to volume expansion and acts on the kidneys to increase dieresis [38]. The association between these two conditions in children is supported by partly or completely resolution of NE after effective treatment of OSA [20], [39].

Nocturnal polyuria has been considered as an important pathogenic factor of NE. This idea was supported by Butler RJ et al. [8]–[9], who noted that a proportion of enuretic children had excessive nocturnal urine production. There is evidence indicating that vitamin D directly contributes to the development of polyuria, which is in agreement with the report that mice lacking the vitamin D receptor (i.e., VDR(−/−) mice) develop polyuria, with 24h urinary volume increased several-fold compared with VDR(+/+) mice [21]. The initial molecular event that leads to the development of polyuria is the upregulation of renin in the kidney and the brain, which is caused by VDR inactivation [40]. The molecular basis for renin upregulation is that 1,25-dihydroxyvitamin D suppresses renin gene transcription by blocking the cAMP response element (CRE)-mediated promoter activity [41]. Renin upregulation leads to an increase in the production of AngII, which, in turn, stimulates the central regulation of water intake, leading to polyuria in a context of normal fluid handling by the kidney [40].

This study has several limitations that should be noted. First, we did not perform a statistical analysis that differentiated between patients with primary and secondary enuresis (i.e., the absence or presence, respectively, of a dry period for over 6 months), however, the majority of children are expected to have primary enuresis. This study also did not differentiate between monosymptomatic and polysymptomatic enuresis (i.e., the absence or presence, respectively, of lower urinary tract dysfunction). Second, family history of bedwetting has been found to significantly affect the prevalence of NE [42], but was not examined in this study.

The article "Relationships between 25-Hydroxyvitamin D and Nocturnal Enuresis in Five- to Seven-Year-Old Children" was published in 2014. Journal: PLoS One.

## Conclusions

In conclusion, this study indicates that there is a statistically significant relationship between serum 25(OH)D concentrations and NE in five- to seven-year-old children. The discovery of the association between 25(OH)D and NE opens a new area of research on the role of vitamin D in the regulation of physiological processes. Further research is needed to confirm this association and to explore more detailed mechanism.

## References

[1] GiovannucciE (2005) The epidemiology of vitamin D and cancer incidence and mortality: a review (United States). Cancer Causes Control 16: 83–95.1586845010.1007/s10552-004-1661-4

[2] NormanAW (2008) From vitamin D to hormone D: fundamentals of the vitamin D endocrine system essential for good health. Am J Clin Nutr 88: 491S–499S.1868938910.1093/ajcn/88.2.491S

[3] Van der SchuerenBJ, VerstuyfA, MathieuC (2012) Straight from D-Heart: vitamin D status and cardiovascular disease. Curr Opin Lipidol 23: 17–23.2212367210.1097/MOL.0b013e32834d7357

[4] GominakSC, StumpfWE (2012) The world epidemic of sleep disorders is linked to vitamin D deficiency. Med Hypotheses 79: 132–135.2258356010.1016/j.mehy.2012.03.031

[5] NeveusT, von GontardA, HoebekeP, HjalmasK, BauerS, et al (2006) The standardization of terminology of lower urinary tract function in children and adolescents: report from the Standardisation Committee of the International Children's Continence Society. J Urol 176: 314–324.1675343210.1016/S0022-5347(06)00305-3

[6] OzdenC, OzdalOL, AltinovaS, OguzulgenI, UrganciogluG, et al (2007) Prevalence and associated factors of enuresis in Turkish children. Int Braz J Urol 33: 216–222.1748854210.1590/s1677-55382007000200013

[7] GumusB, VurgunN, LekiliM, IscanA, MuezzinogluT, et al (1999) Prevalence of nocturnal enuresis and accompanying factors in children aged 7–11 years in Turkey. Acta Paediatr 88: 1369–1372.1062652410.1080/080352599750030103

[8] ButlerRJ (2004) Childhood nocturnal enuresis: developing a conceptual framework. Clin Psychol Rev 24: 909–931.1553327810.1016/j.cpr.2004.07.001

[9] ButlerRJ, HollandP (2000) The three systems: a conceptual way of understanding nocturnal enuresis. Scand J Urol Nephrol 34: 270–277.1109508710.1080/003655900750042022

[10] RoehrsT, MerlottiL, PetrucelliN, StepanskiE, RothT (1994) Experimental sleep fragmentation. Sleep 17: 438–443.799195510.1093/sleep/17.5.438

The article "Relationships between 25-Hydroxyvitamin D and Nocturnal Enuresis in Five- to Seven-Year-Old Children" was published in 2014. Journal: PLoS One.

[11] EylesDW, SmithS, KinobeR, HewisonM, McGrathJJ (2005) Distribution of the vitamin D receptor and 1 alpha-hydroxylase in human brain. J Chem Neuroanat 29: 21–30.1558969910.1016/j.jchemneu.2004.08.006

[12] HuangW, ShahS, LongQ, CrankshawAK, TangprichaV (2013) Improvement of pain, sleep, and quality of life in chronic pain patients with vitamin D supplementation. Clin J Pain 29: 341–347.2269914110.1097/AJP.0b013e318255655d

[13] McCartyDE (2010) Resolution of hypersomnia following identification and treatment of vitamin d deficiency. J Clin Sleep Med 6: 605–608.21206551PMC3014249

[14] AbuzeidWM, AkbarNA, ZacharekMA (2012) Vitamin D and chronic rhinitis. Curr Opin Allergy Clin Immunol 12: 13–17.2219305210.1097/ACI.0b013e32834eccdb

[15] NunnJD, KatzDR, BarkerS, FraherLJ, HewisonM, et al (1986) Regulation of human tonsillar T-cell proliferation by the active metabolite of vitamin D3. Immunology 59: 479–484.3026959PMC1453330

[16] ReidD, MortonR, SalkeldL, BartleyJ (2011) Vitamin D and tonsil disease—preliminary observations. Int J Pediatr Otorhinolaryngol 75: 261–264.2113106410.1016/j.ijporl.2010.11.012

[17] GlerupH, MikkelsenK, PoulsenL, HassE, OverbeckS, et al (2000) Hypovitaminosis D myopathy without biochemical signs of osteomalacic bone involvement. Calcif Tissue Int 66: 419–424.1082187710.1007/s002230010085

[18] PrabhalaA, GargR, DandonaP (2000) Severe myopathy associated with vitamin D deficiency in western New York. Arch Intern Med 160: 1199–1203.1078961510.1001/archinte.160.8.1199

[19] RussellJA (1994) Osteomalacic myopathy. Muscle Nerve 17: 578–580.819669910.1002/mus.880170603

[20] UmlaufMG, ChasensER (2003) Bedwetting—not always what it seems: a sign of sleep-disordered breathing in children. J Spec Pediatr Nurs 8: 22–30.1271540310.1111/j.1744-6155.2003.tb00180.x

[21] LiYC, KongJ, WeiM, ChenZF, LiuSQ, et al (2002) 1,25-Dihydroxyvitamin D(3) is a negative endocrine regulator of the renin-angiotensin system. J Clin Invest 110: 229–238.1212211510.1172/JCI15219PMC151055

[22] van den OuwelandJM, VogeserM, BacherS (2013) Vitamin D and metabolites measurement by tandem mass spectrometry. Rev Endocr Metab Disord 14: 159–184.2353948410.1007/s11154-013-9241-0

[23] HolickMF, BinkleyNC, Bischoff-FerrariHA, GordonCM, HanleyDA, et al (2011) Evaluation, treatment, and prevention of vitamin D deficiency: an Endocrine Society clinical practice guideline. J Clin Endocrinol Metab 96: 1911–1930.2164636810.1210/jc.2011-0385

[24] RossAC, MansonJE, AbramsSA, AloiaJF, BrannonPM, et al (2011) The 2011 report on dietary reference intakes for calcium and vitamin D from the Institute of Medicine: what clinicians need to know. J Clin Endocrinol Metab 96: 53–58.2111882710.1210/jc.2010-2704PMC3046611

The article "Relationships between 25-Hydroxyvitamin D and Nocturnal Enuresis in Five- to Seven-Year-Old Children" was published in 2014. Journal: PLoS One.

[25] SaintongeS, BangH, GerberLM (2009) Implications of a new definition of vitamin D deficiency in a multiracial us adolescent population: the National Health and Nutrition Examination Survey III. Pediatrics 123: 797–803.1925500510.1542/peds.2008-1195

[26] NeveusT (2008) Enuretic sleep: deep, disturbed or just wet? Pediatr Nephrol 23: 1201–1202.1848110610.1007/s00467-008-0859-1

[27] Cohen-ZrubavelV, KushnirB, KushnirJ, SadehA (2011) Sleep and sleepiness in children with nocturnal enuresis. Sleep 34: 191–194.2128625210.1093/sleep/34.2.191PMC3022939

[28] PhilipP, StoohsR, GuilleminaultC (1994) Sleep fragmentation in normals: a model for sleepiness associated with upper airway resistance syndrome. Sleep 17: 242–247.7939124

[29] KiddooDA, ValentinoRJ, ZdericS, GaneshA, LeiserSC, et al (2006) Impact of state of arousal and stress neuropeptides on urodynamic function in freely moving rats. Am J Physiol Regul Integr Comp Physiol 290: R1697–1706.1643966710.1152/ajpregu.00742.2005

[30] SuzukiY, IchiyamaT, OhsakiA, HasegawaS, ShiraishiM, et al (2009) Anti-inflammatory effect of 1alpha,25-dihydroxyvitamin D(3) in human coronary arterial endothelial cells: Implication for the treatment of Kawasaki disease. J Steroid Biochem Mol Biol 113: 134–138.1913873910.1016/j.jsbmb.2008.12.004

[31] JablonskiKL, ChoncholM, PierceGL, WalkerAE, SealsDR (2011) 25-Hydroxyvitamin D deficiency is associated with inflammation-linked vascular endothelial dysfunction in middle-aged and older adults. Hypertension 57: 63–69.2111587810.1161/HYPERTENSIONAHA.110.160929PMC3020150

[32] KruegerJM, MajdeJA, RectorDM (2011) Cytokines in immune function and sleep regulation. Handb Clin Neurol 98: 229–240.2105619010.1016/B978-0-444-52006-7.00015-0PMC5440845

[33] PetersonCA, HeffernanME (2008) Serum tumor necrosis factor-alpha concentrations are negatively correlated with serum 25(OH)D concentrations in healthy women. J Inflamm (Lond) 5: 10.1865268010.1186/1476-9255-5-10PMC2503979

[34] VgontzasAN, ZoumakisE, LinHM, BixlerEO, TrakadaG, et al (2004) Marked decrease in sleepiness in patients with sleep apnea by etanercept, a tumor necrosis factor-alpha antagonist. J Clin Endocrinol Metab 89: 4409–4413.1535603910.1210/jc.2003-031929

[35] McCartyDE, ReddyA, KeigleyQ, KimPY, MarinoAA (2012) Vitamin D, race, and excessive daytime sleepiness. J Clin Sleep Med 8: 693–697.2324340310.5664/jcsm.2266PMC3501666

[36] LeibermanA, Stiller-TimorL, TarasiukA, TalA (2006) The effect of adenotonsillectomy on children suffering from obstructive sleep apnea syndrome (OSAS): the Negev perspective. Int J Pediatr Otorhinolaryngol 70: 1675–1682.1685447110.1016/j.ijporl.2006.06.002

The article "Relationships between 25-Hydroxyvitamin D and Nocturnal Enuresis in Five- to Seven-Year-Old Children" was published in 2014. Journal: PLoS One.

[37] BeebeDW (2006) Neurobehavioral morbidity associated with disordered breathing during sleep in children: a comprehensive review. Sleep 29: 1115–1134.1704000010.1093/sleep/29.9.1115

[38] BrennerBM, BallermannBJ, GunningME, ZeidelML (1990) Diverse biological actions of atrial natriuretic peptide. Physiol Rev 70: 665–699.214194410.1152/physrev.1990.70.3.665

[39] HjalmasK, ArnoldT, BowerW, CaioneP, ChiozzaLM, et al (2004) Nocturnal enuresis: an international evidence based management strategy. J Urol 171: 2545–2561.10.1097/01.ju.0000111504.85822.b215118418

[40] KongJ, ZhangZ, LiD, WongKE, ZhangY, et al (2008) Loss of vitamin D receptor produces polyuria by increasing thirst. J Am Soc Nephrol 19: 2396–2405.1883243810.1681/ASN.2008010011PMC2588110

[41] YuanW, PanW, KongJ, ZhengW, SzetoFL, et al (2007) 1,25-dihydroxyvitamin D3 suppresses renin gene transcription by blocking the activity of the cyclic AMP response element in the renin gene promoter. J Biol Chem 282: 29821–29830.1769009410.1074/jbc.M705495200

[42] GunesA, GunesG, AcikY, AkilliA (2009) The epidemiology and factors associated with nocturnal enuresis among boarding and daytime school children in southeast of Turkey: a cross sectional study. BMC Public Health 9: 357.1977265710.1186/1471-2458-9-357PMC2754466

